The article "On Suitability of Mixture of Generalized Exponential Models in Modeling Right-Censored Medical Datasets Using Conditional Expectations" was published in 2022. Journal: Comput Math Methods Med.

# On Suitability of Mixture of Generalized Exponential Models in Modeling Right-Censored Medical Datasets Using Conditional Expectations

**DOI:** 10.1155/2022/7363646

**Published:** 2022-10-14

**Authors:** Navid Feroze, Ali Akgül, Ali A. Al-Alwan, Md. Moyazzem Hossain, R. Alshenawy

**Affiliations:** ^1^Department of Statistics, The University of Azad Jammu and Kashmir, Muzaffarabad, Pakistan; ^2^Art and Science Faculty, Department of Mathematics, Siirt University, 56100 Siirt, Turkey; ^3^Mathematics Research Center, Department of Mathematics, Near East University, Near East Boulevard, PC: 99138 Nicosia /Mersin 10, Turkey; ^4^Department of Mathematics and Statistics, College of Science, King Faisal University, P. O. Box 400, Al-Ahsa 31982, Saudi Arabia; ^5^Department of Statistics, Jahangirnagar University, Savar, Dhaka 1342, Bangladesh; ^6^Department of Applied Statistics and Insurance, Faculty of Commerce, Mansoura University, Mansoura 35516, Egypt

## Abstract

The exploration of suitable models for modeling censored medical datasets is of great importance. There are numerous studies dealing with modeling the censored medical datasets. However, majority of the earlier contributions have utilized the conventional models for modeling the said datasets. Unfortunately, the conventional models are not capable of capturing the behavior of the heterogeneous datasets involving the mixture of two or more subpopulations. In addition, the earlier contributions have considered conventional censoring schemes by replacing all the censored items with the largest failed item. This paper is aimed at proposing the analysis of right-censored mixture medical datasets. The mixture of the generalized exponential distribution has been proposed to model the right-censored heterogeneous medical datasets. In converse to conventional censoring schemes, we have proposed censoring schemes which replace the censored items with conditional expectation (CE) of the random variable. In addition, the Bayesian methods have been proposed to estimate the model parameters. The performance and sensitivity of the proposed estimators have been evaluated using a detailed simulation study. The detailed simulation study suggests that censoring schemes based on CE provide improved estimation as compared to conventional censoring schemes. The suitability of the model in modeling heterogeneous datasets has been verified by modeling two real right-censored medical datasets. The comparison of the proposed model with existing mixture model under Bayesian methods advocated the improved performance of the proposed model.

## 1. Introduction

The exploration of suitable models for modeling censored medical datasets is of great importance. There are numerous studies dealing with modeling the censored medical datasets. However, majority of the earlier contributions have utilized the conventional models for modeling the said datasets. Unfortunately, the conventional models are not capable of capturing the behavior of the heterogeneous datasets involving the mixture of two or more subpopulations. Some researchers have considered mixture models for analysis of medical datasets. Hanson [1] proposed mixture of Gamma distributions to model the survival times of the lung cancer patients. Noor et al. [2] considered the mixture of exponential models to analyze the data regarding incidents of mortality due the different types of the cancer. Bussy et al. [3] introduced a supervised learning mixed model for modeling censored mixture data. The estimation of the model parameters was carried out using Expectation Maximization (EM) algorithm. The applicability of the proposed model was illustrated using three real datasets relating to genetic cancer. Mahmud et al. [4] proposed a mixture of log-skew-normal distributions for analysis of data from a Diary of Asthma and Viral Infectious Study conducted during 2004. Geissen et al. [5] presented multiexperiment mixture model that enables the researchers to simultaneously model censored and uncensored data. Cheung et al. [6] proposed a family of mixture models for undiagnosed prevalent disease with interval-censored incidents. Xiang et al. [7] proposed a mixture cure model for analysis of the survival data with a cure fraction. The estimation under the proposed model was carried out using EM algorithm. However, earlier contributions regarding analysis of censored mixture medical data have utilized the classical method of estimation, such as maximum likelihood estimation and EM algorithm. Recently, Noor et al. [2] proposed Bayesian methods for analysis of heterogeneous medical datasets. However, the model proposed by Noor et al. [2] was less flexible as it has no shape parameters. Resultantly, the corresponding analysis was quite straight forward. In addition, all of the above contributions have considered conventional censoring environment which replaces the censored items either by test termination time (for type-I censoring) or by the largest observed value (for type-II censoring). In other words, the censored items have been simply replaced by a common predetermined value. Statistical properties of estimates based on such censoring environment can be unclear [8]. Steiner and Mackay [9] addressed this issue by proposing the use of conditional expectation (CE) of random variable as a replacement for the censored items. However, the said proposal was for the single models. A careful review of literature suggests that the use of CE has never been considered for the censored mixture models.

The article "On Suitability of Mixture of Generalized Exponential Models in Modeling Right-Censored Medical Datasets Using Conditional Expectations" was published in 2022. Journal: Comput Math Methods Med.

The generalized exponential distribution (GED) is very important lifetime distribution. It has more features as compared to exponential and Rayleigh distribution as it has the shape parameter. The utilization of GED is convenient as compared to lognormal and gamma distribution as it has closed form expressions for cumulative distribution function and the hazard rate function. Few studies have also concluded that the performance of GED is better as compared to Weibull distribution in modeling censored data [10]. The mixture of GED (MGED) has been introduced more recently. The analysis of MGED under progressive censoring was considered by Wang et al. [11]. Teng and Zhang [12] showed that the Gaussian mixture and Laplacian mixture can be obtained as special cases of MGED. The estimation of model parameters was considered using EM algorithm. The superiority of MGED over Weibull distribution was explored by Ateya [13], and the industrial applications of MGED were reported by Ali et al. [14]. Mohamed et al. [15] introduced the methodology to obtain the Bayesian predictions using MGED. Kazmi and Aslam [16] considered the Bayesian analysis for right censored using MGED assuming shape parameters to be known. The above discussion suggests that the MGED is very relevant distribution in modeling the censored datasets. However, the suitability of MGED in modeling right-censored mixture datasets from medical fields using Bayesian methods is still to be explored.

We have considered the Bayesian estimation of two-component MGED (2CMGED) when samples are right censored. The applicability of the proposed model in modeling right-censored heterogeneous datasets from medical sciences has been explored using real datasets. The main feature of the paper is the introduction of censoring environment in which the censored items are replaced by the CE of the random variable. We have compared the proposed censoring environment with the existing censoring environment in which the censored items are replaced by the largest observed value. The Bayesian estimation has been carried out assuming noninformative (NIP) and informative priors (IP). Four loss functions, namely, squared error loss function (SELF), precautionary loss function (PLF), entropy loss function (ELF) and, LINEX loss function (LLF) have been used for the analysis. Since the Bayesian estimates (BEs) were unavailable in closed form, the Bayesian approximate methods, namely, Lindley's approximation (LA) and importance sampling (IS) were used for the numerical computations. The performance of the proposed model was compared with two-component mixture of exponential distribution (2CMED). The said comparison advocated the superiority of the 2CMGED over 2CMED. In addition, the results based on proposed CE censoring environment provided improved estimation as compared to conventional censoring environment.

The article "On Suitability of Mixture of Generalized Exponential Models in Modeling Right-Censored Medical Datasets Using Conditional Expectations" was published in 2022. Journal: Comput Math Methods Med.

## 2. Materials and Methods

The probability density function (PDF) of the generalized exponential distribution is

(1) $$\begin{array}{c} f_{j}\left(x_{j};\lambda_{j},\theta_{j}\right)=\lambda_{j}\theta_{j}{\left(1-e^{-\theta_{j}x_{j}}\right)}^{\lambda_{j}-1}e^{-\theta_{j}x_{j}},\;0<x_{j}<\infty ,\;\lambda_{j},\theta_{j}>0,\;j=1,2, \end{array}$$

where *X*_*j*_ is random variable and *λ*_*j*_ and *θ*_*j*_ are the parameters of the distribution.

The CDF of the generalized exponential distribution is

(2) $$\begin{array}{c} F_{j}\left(x_{j};\lambda_{j},\theta_{j}\right)={\left(1-e^{-\theta_{j}x_{j}}\right)}^{\lambda_{j}},\;0<x_{j}<\infty ,\;\lambda_{j},\theta_{j}>0,\;j=1,2. \end{array}$$

The two-component mixture of generalized exponential distributions (2CMGED) with mixing weights (*π*_1_,*π*_2_ = 1 − *π*_1_) is

(3) $$\begin{array}{c} f\left(x;\Omega \right)=\overset{2}{\underset{u=1}{\sum }}\pi_{u}\lambda_{u}\theta_{u}{\left(1-e^{-\theta_{u}x_{u}}\right)}^{\lambda_{u}-1}e^{-\theta_{u}x_{u}},\;0<x_{u}<\infty , \end{array}$$

where **Ω** = (*λ*_1_, *λ*_2_, *θ*_1_, *θ*_2_, *π*_1_); 0 < *π*_1_ < 1; *λ*_*u*_, *θ*_*u*_ > 0.

The cumulative distribution function for the 2CMGED is

(4) $$\begin{array}{c} F\left(x;\Omega \right)=\overset{2}{\underset{u=1}{\sum }}\pi_{u}{\left(1-e^{-\theta_{u}x}\right)}^{\lambda_{u}},\;0<x_{u}<\infty . \end{array}$$

### 2.1. Bayesian Estimation under Right-Censored Samples

In this section, the right-censored samples have been used to estimate the parameters of 2CMGED. Unfortunately, the proposed BEs do not exist in the explicit form; hence the approximate Bayesian methods have been used for the estimation.

#### 2.1.1. The Likelihood Function under Right-Censored Samples

Consider a sample of size ‘*n*' from 2CMGED from which *n*_1_ = *π*_1_*n* and *n*_2_ = (1 − *π*_1_)*n* number of observation are assumed to come from component-I and component-II of the mixture. Suppose *r*_1_ and *r*_2_ number of failed items observed from component-I and component-II, respectively. The remaining *n*_1_ − *r*_1_ and *n*_2_ − *r*_2_ items have been assumed to be censored from each component. Then the likelihood function for such right-censored mixture data can be written as

(5) $$\begin{array}{c} l\left(\Omega ;x\right)\propto \overset{r_{1}}{\underset{i=1}{\prod }}\pi_{1}f_{1}\left(x_{1i}\right)\overset{r_{2}}{\underset{i=1}{\prod }}\left(1-\pi_{1}\right)f_{2}\left(x_{2i}\right){\left[1-F\left(x_{r}\right)\right]}^{n-r}, \end{array}$$

where *r* = *r*_1_ + *r*_2_, *x*_*r*_ = max(*x*_*r*1_, *x*_*r*2_) is an order statistic.

The article "On Suitability of Mixture of Generalized Exponential Models in Modeling Right-Censored Medical Datasets Using Conditional Expectations" was published in 2022. Journal: Comput Math Methods Med.

Putting the results in Equation (5), we have

(6) $$\begin{array}{c} \begin{array}{c} l\left(\Omega \left|x\right.\right)=\pi_{1}^{r_{1}}{\left(1-\pi_{1}\right)}^{r_{2}}\lambda_{1}^{r_{1}}\theta_{1}^{r_{1}}\lambda_{2}^{r_{2}}\theta_{2}^{r_{2}}\exp\left\{\left(\lambda_{1}-1\right)\overset{r_{1}}{\underset{i=1}{\sum }}\log\left(1-e^{-\theta_{1}x_{1i}}\right)\right\}\exp\left\{\left(\lambda_{2}-1\right)\overset{r_{2}}{\underset{i=1}{\sum }}\log\left(1-e^{-\theta_{2}x_{2i}}\right)\right\}\\ \;\times e^{-\theta_{1}\overset{r_{1}}{\underset{i=1}{\sum }}x_{1i}}e^{-\theta_{2}\overset{r_{2}}{\underset{i=1}{\sum }}x_{2i}}{\left\{1-\pi_{1}{\left(1-e^{-\theta_{1}t}\right)}^{\lambda_{1}}-\left(1-\pi_{1}\right){\left(1-e^{-\theta_{1}t}\right)}^{\lambda_{2}}\right\}}^{n-r}. \end{array} \end{array}$$

The conventional censoring schemes replace the censored items by the largest observed value. This assumption is not suitable because the censoring items are surely greater than the largest observed value. The appropriate solution to this issue is to replace the censored items with CE of the random variable. The conditional distribution for model given in Equation (1) is

(7) $$\begin{array}{c} f\left(X_{j}\left|X_{j}>x_{j}\right.\right)=\frac{\lambda_{j}\theta_{j}{\left(1-e^{-\theta_{j}x_{j}}\right)}^{\lambda_{j}-1}e^{-\theta_{j}x_{j}}}{1-{\left(1-e^{-\theta_{j}x_{j}}\right)}^{\lambda_{j}}}. \end{array}$$

The CE for Equation (1) is

(8) $$\begin{array}{c} Ε\left(X_{j}\left|X_{j}>x_{r}\right.\right)=\lambda_{j}\theta_{j}\int_{x_{r}}^{\infty }x_{j}{\left(1-e^{-\theta_{j}x_{j}}\right)}^{\lambda_{j}-1}e^{-\theta_{j}x_{j}}{dx}_{j}. \end{array}$$

Since the analytical solutions for CE are not possible. The values for CE have been obtained numerically using numerical integrations.

So, the resulting dataset is of the form

(9) $$\begin{array}{c} X_{ij}=\left\{\begin{array}{c} x_{ij}\text{ for observed items}\\ CE\text{ for censored items} \end{array}\right.. \end{array}$$

#### 2.1.2. Priors and Posterior Distributions

We have proposed two sets of priors for the parameters of the 2CMGED. One set contains the NIP, while the other set is the combination of IPs. The description of each set of priors is presented in the followings.

The combined NIP for the parametric set **Ω** is

(10) $$\begin{array}{c} h_{1}\left(\Omega \right)\propto 1,\;\lambda_{1},\lambda_{2},\theta_{1},\theta_{2}>0,\;0<\pi_{1}<1, \end{array}$$

where the model parameters have uniform priors over the rage (0, 1).

The article "On Suitability of Mixture of Generalized Exponential Models in Modeling Right-Censored Medical Datasets Using Conditional Expectations" was published in 2022. Journal: Comput Math Methods Med.

Based on NIP given in Equation (10), the posterior distribution for **Ω** is

(11) $$\begin{array}{c} \begin{array}{c} g_{1}\left(\Omega \left|x\right.\right)\propto \pi_{1}^{r_{1}}{\left(1-\pi_{1}\right)}^{r_{2}}\overset{2}{\underset{u=1}{\prod }}\lambda_{u}^{r_{u}}\theta_{u}^{r_{u}}\exp\left\{\left(\lambda_{u}-1\right)\overset{r_{u}}{\underset{i=1}{\sum }}\log\left(1-e^{-\theta_{u}x_{ui}}\right)\right\}\\ \times e^{-\theta_{u}\overset{r_{u}}{\underset{i=1}{\sum }}x_{ui}}{\left\{1-\pi_{1}{\left(1-e^{-\theta_{1}t}\right)}^{\lambda_{1}}-\left(1-\pi_{1}\right){\left(1-e^{-\theta_{1}t}\right)}^{\lambda_{2}}\right\}}^{n-r}. \end{array} \end{array}$$

Again, let *π*_1_ ~ Beta(*a*_1_, *b*_1_), *λ*_*u*_ ~ Gamma(*a*_1*u*_, *b*_1*u*_)_,_ and *θ*_*u*_ ~ Gamma(*a*_2*u*_, *b*_2*u*_), where

*a*_1_, *b*_1_, *a*_1*u*_, *b*_1*u*_, *a*_2*u*_, *b*_2*u*_ > 0, *u* = 1, 2 are the hyperparameters.

Then, the combined prior distribution for **Ω**is

(12) $$\begin{array}{c} h_{2}\left(\Omega \right)\propto \pi_{1}^{a_{1}-1}{\left(1-\pi_{1}\right)}^{b_{1}-1}\overset{2}{\underset{u=1}{\prod }}\lambda_{u}^{a_{2u}-1}\exp\left(-b_{2u}\lambda_{u}\right)\theta_{u}^{a_{3u}-1}\exp\left(-b_{3u}\theta_{u}\right),0<\pi_{1}<1,\lambda_{u},\beta_{u}>0. \end{array}$$

The posterior distribution under Equation (12) is

(13) $$\begin{array}{c} \begin{array}{c} g_{2}\left(\Omega \left|x\right.\right)\propto \pi_{1}^{r_{1}+a_{1}-1}{\left(1-\pi_{1}\right)}^{r_{2}+b_{1}-1}\overset{2}{\underset{u=1}{\prod }}\lambda_{u}^{r_{u}+a_{1u}-1}\theta_{u}^{r_{u}+a_{2u}-1}\exp\left\{\left(\lambda_{u}-1\right)\overset{r_{u}}{\underset{i=1}{\sum }}\log\left(1-e^{-\theta_{u}x_{ui}}\right)-\lambda_{u}b_{1u}\right\}\\ \times e^{-\theta_{u}\left(\overset{r_{u}}{\underset{i=1}{\sum }}x_{ui}+b_{2u}\right)}{\left\{1-\pi_{1}{\left(1-e^{-\theta_{1}t}\right)}^{\lambda_{1}}-\left(1-\pi_{1}\right){\left(1-e^{-\theta_{1}t}\right)}^{\lambda_{2}}\right\}}^{n-r}. \end{array} \end{array}$$

As the posterior distributions under both priors do not provide closed form estimators, we have proposed approximate estimation in the coming sections.

#### 2.1.3. Lindley's Approximation (LA)

This section considers the LA for approximate solution of the model parameters. If sample size is sufficiently large, then according to Lindley, any ratio of the integrals of the form

(14) $$\begin{array}{c} I\left(\Omega \right)=Ε\left[w\left(\Omega \right)\right]=\frac{\int_{\Omega }w\left(\Omega \right)\exp\left\{L\left(\Omega ;x\right)+H\left(\Omega \right)\right\}d\Omega }{\int_{\Omega }\exp\left\{L\left(\Omega ;x\right)+H\left(\Omega \right)\right\}d\Omega }, \end{array}$$

where *w*(**Ω**) is any function of *λ*_1_, *λ*_2_, *θ*_1_, *θ*_2_, *π*_1_, *L*(**Ω**|**x**) is the log-likelihood function and *H*(**Ω**) is the logarithmic of joint prior for the parametric set **Ω**, can be evaluated as

(15) $$\begin{array}{c} \begin{array}{c} I\left(\Omega \right)=w\left(\hat{\Omega }\right)+\left(g_{1}d_{1}+g_{2}d_{2}+g_{3}d_{3}+g_{4}d_{4}+g_{5}d_{5}+d_{6}+d_{7}\right)\\ +\frac{1}{2}\left(A_{1}B_{1}+A_{2}B_{2}+A_{3}B_{3}+A_{4}B_{4}+A_{5}B_{5}\right), \end{array} \end{array}$$

where $\hat{\Omega }$is the maximum likelihood estimator (MLE) of the parametric set **Ω**.

(16) $$\begin{array}{c} B_{i}=g_{1}\sigma_{i1}+g_{2}\sigma_{i2}+g_{3}\sigma_{i3}+g_{4}\sigma_{i4}+g_{5}\sigma_{i5}, \end{array}$$

(17) $$\begin{array}{c} \begin{array}{c} A_{i}=\sigma_{11}L_{11i}+\sigma_{22}L_{22i}+\sigma_{33}L_{33i}+\sigma_{44}L_{44i}+\sigma_{55}L_{55i}+2\sigma_{12}L_{12i}+2\sigma_{13}L_{13i}+2\sigma_{14}L_{14i}+2\sigma_{15}L_{15i}\\ +2\sigma_{23}L_{23i}+2\sigma_{24}L_{24i}+2\sigma_{25}L_{25i}+2\sigma_{34}L_{34i}+2\sigma_{35}L_{35i}+2\sigma_{45}L_{45i}, \end{array} \end{array}$$

(18) $$\begin{array}{c} d_{i}=P_{1}\sigma_{i1}+P_{2}\sigma_{i2}+P_{3}\sigma_{i3}+P_{4}\sigma_{i4}+P_{5}\sigma_{i5},\;i=1,2,3,4,5, \end{array}$$

(19) $$\begin{array}{c} d_{6}=g_{12}\sigma_{12}+g_{13}\sigma_{13}+g_{14}\sigma_{14}+g_{15}\sigma_{15}+g_{23}\sigma_{23}+g_{24}\sigma_{24}+g_{25}\sigma_{25}+g_{34}\sigma_{34}+g_{35}\sigma_{35}+g_{45}\sigma_{45}, \end{array}$$

(20) $$\begin{array}{c} d_{7}=\frac{1}{2}\left(g_{11}\sigma_{11}+g_{22}\sigma_{22}+g_{33}\sigma_{33}+g_{44}\sigma_{44}+g_{55}\sigma_{55}\right), \end{array}$$

(21) $$\begin{array}{c} P_{i}=\frac{\partial H\left(\Omega \right)}{\partial \Omega_{i}},\;i=1,2,3,4,5,\;g_{ij}=\frac{\partial^{2}w\left(\Omega \right)}{\partial \Omega_{i}\partial \Omega_{j}},\;L_{ij}=\frac{\partial^{2}L\left(\Omega \left|x\right.\right)}{\partial \Omega_{i}\partial \Omega_{j}},\;i,j=1,2,3,4,5, \end{array}$$

(22) $$\begin{array}{c} L_{ijk}=\frac{\partial^{3}L_{11}\left(\Omega_{11}\left|x\right.\right)}{\partial \Omega_{11i}\partial \Omega_{11j}\partial \Omega_{11k}},\;i,j,k=1,2,3,4,5, \end{array}$$

where *S*_*ij*_is the (*i*, *j*)^*th*^ element of the inverse of the matrix {*L*_*ij*_}, all evaluated at the MLEs of the parameters.

The article "On Suitability of Mixture of Generalized Exponential Models in Modeling Right-Censored Medical Datasets Using Conditional Expectations" was published in 2022. Journal: Comput Math Methods Med.

The log-likelihood function from Equation (6) is

(23) $$\begin{array}{c} \begin{array}{c} L\left(\Omega ;x\right)=r_{1}\log\pi_{1}+r_{2}\log\left(1-\pi_{1}\right)+r_{1}\log\lambda_{1}+r_{2}\log\lambda_{2}+r_{1}\log\theta_{1}+r_{2}\log\theta_{2}\\ -\theta_{1}\overset{r_{1}}{\underset{i=1}{\sum }}x_{1i}-\theta_{2}\overset{r_{2}}{\underset{i=1}{\sum }}x_{2i}+\left(\lambda_{1}-1\right)\overset{r_{1}}{\underset{i=1}{\sum }}\log\left(1-e^{-\theta_{1}x_{1i}}\right)+\left(\lambda_{2}-1\right)\overset{r_{2}}{\underset{i=1}{\sum }}\log\left(1-e^{-\theta_{2}x_{2i}}\right)\\ +\left(n-r\right)\log\left\{1-\pi_{1}{\left(1-e^{-\theta_{1}t}\right)}^{\lambda_{1}}-\left(1-\pi_{1}\right){\left(1-e^{-\theta_{1}t}\right)}^{\lambda_{2}}\right\}. \end{array} \end{array}$$

The MLEs of the parameters are obtained by iterative solution of the following:

(24) $$\begin{array}{c} \frac{r_{1}}{\lambda_{1}}-\frac{\left(n-r\right)\pi_{1}{\left(1-e^{-\theta_{1}t}\right)}^{\lambda_{1}}\log\left(1-e^{-\theta_{1}t}\right)}{F\left(t;\Omega_{13}\right)}+\overset{r_{1}}{\underset{i=1}{\sum }}\log\left(1-e^{-\theta_{1}x_{1i}}\right)=0, \end{array}$$

(25) $$\begin{array}{c} \frac{r_{2}}{\lambda_{2}}-\frac{\left(n-r\right)\left(1-\pi_{1}\right){\left(1-e^{-\theta_{2}t}\right)}^{\lambda_{2}}\log\left(1-e^{-\theta_{2}t}\right)}{F\left(t;\Omega_{13}\right)}+\overset{r_{2}}{\underset{i=1}{\sum }}\log\left(1-e^{-\theta_{2}x_{2i}}\right)=0, \end{array}$$

(26) $$\begin{array}{c} \frac{r_{1}}{\theta_{1}}-\frac{\left(n-r\right)\pi_{1}\lambda_{1}{te}^{-\theta_{1}t}{\left(1-e^{-\theta_{1}t}\right)}^{\lambda_{1}-1}}{F\left(t;\Omega_{13}\right)}-\overset{r_{1}}{\underset{i=1}{\sum }}x_{1i}+\left(\lambda_{1}-1\right)\overset{r_{1}}{\underset{i=1}{\sum }}\frac{x_{1i}e^{-\theta_{1}x_{1i}}}{1-e^{-\theta_{1}x_{1i}}}=0, \end{array}$$

(27) $$\begin{array}{c} \frac{r_{2}}{\theta_{2}}-\frac{\left(n-r\right)\left(1-\pi_{1}\right)\lambda_{2}{te}^{-\theta_{2}t}{\left(1-e^{-\theta_{2}t}\right)}^{\lambda_{2}-1}}{F\left(t;\Omega_{13}\right)}-\overset{r_{2}}{\underset{i=1}{\sum }}x_{2i}+\left(\lambda_{2}-1\right)\overset{r_{2}}{\underset{i=1}{\sum }}\frac{x_{2i}e^{-\theta_{2}x_{2i}}}{1-e^{-\theta_{2}x_{2i}}}=0, \end{array}$$

(28) $$\begin{array}{c} \frac{r_{1}}{\pi_{1}}-\frac{r_{2}}{1-\pi_{1}}-\frac{\left(n-r\right)\left\{{\left(1-e^{-\theta_{2}t}\right)}^{\lambda_{2}}-{\left(1-e^{-\theta_{1}t}\right)}^{\lambda_{1}}\right\}}{F\left(t;\Omega_{13}\right)}=0. \end{array}$$

The MLEs for the parametric set **Ω** is denoted by $\hat{\Omega }=\left({\hat{\lambda }}_{1},{\hat{\lambda }}_{2},{\hat{\theta }}_{1},{\hat{\theta }}_{2},{\hat{\pi }}_{1}\right)$. As mentioned in the previous sections, the second order and third order derivatives from the Equation ((13) have not been presented here. Based on the second order derivatives, the elements of the matrix {*L*_*ij*_}^−1^ are obtained and denoted by *σ*_*ij*_, where *i*, *j* = 1, 2, 3, 4, 5.

Using LA, the BEs for **Ω**, under SELF and NIP, are given in the following:

(29) $$\begin{array}{c} \theta_{1,\text{SELF}}={\hat{\theta }}_{1}+\frac{1}{2}\left(A_{1}\sigma_{11}+A_{2}\sigma_{21}+A_{3}\sigma_{31}+A_{4}\sigma_{41}+A_{5}\sigma_{51}\right), \end{array}$$

(30) $$\begin{array}{c} \theta_{2,\text{SELF}}={\hat{\theta }}_{2}+\frac{1}{2}\left(A_{1}\sigma_{12}+A_{2}\sigma_{22}+A_{3}\sigma_{32}+A_{4}\sigma_{42}+A_{5}\sigma_{52}\right), \end{array}$$

(31) $$\begin{array}{c} \lambda_{1,\text{SELF}}={\hat{\lambda }}_{1}+\frac{1}{2}\left(A_{1}\sigma_{13}+A_{2}\sigma_{23}+A_{3}\sigma_{33}+A_{4}\sigma_{43}+A_{5}\sigma_{53}\right), \end{array}$$

(32) $$\begin{array}{c} \lambda_{2,\text{SELF}}={\hat{\lambda }}_{2}+\frac{1}{2}\left(A_{1}\sigma_{14}+A_{2}\sigma_{24}+A_{3}\sigma_{34}+A_{4}\sigma_{44}+A_{5}\sigma_{54}\right), \end{array}$$

(33) $$\begin{array}{c} \pi_{1,\text{SELF}}={\hat{\pi }}_{1}+\frac{1}{2}\left(A_{1}\sigma_{15}+A_{2}\sigma_{25}+A_{3}\sigma_{35}+A_{4}\sigma_{45}+A_{5}\sigma_{55}\right). \end{array}$$

Similarly considering LA, the BEs for **Ω**, under SELF and NIP are

(34) $$\begin{array}{c} \theta_{1,\text{PLF}}=\sqrt{{\hat{\theta }}_{1}^{2}+\frac{1}{2}\left(2{\hat{\theta }}_{1}\sigma_{11}+A_{1}\sigma_{11}+A_{2}\sigma_{21}+A_{3}\sigma_{31}+A_{4}\sigma_{41}+A_{5}\sigma_{51}\right)}, \end{array}$$

(35) $$\begin{array}{c} \theta_{2,\text{PLF}}=\sqrt{{\hat{\theta }}_{2}^{2}+\frac{1}{2}\left(2{\hat{\theta }}_{2}\sigma_{22}+A_{1}\sigma_{12}+A_{2}\sigma_{22}+A_{3}\sigma_{32}+A_{4}\sigma_{42}+A_{5}\sigma_{52}\right)}, \end{array}$$

(36) $$\begin{array}{c} \lambda_{1,\text{PLF}}=\sqrt{{\hat{\lambda }}_{1}^{2}+\frac{1}{2}\left(2{\hat{\lambda }}_{1}\sigma_{33}+A_{1}\sigma_{13}+A_{2}\sigma_{23}+A_{3}\sigma_{33}+A_{4}\sigma_{43}+A_{5}\sigma_{53}\right)}, \end{array}$$

(37) $$\begin{array}{c} \lambda_{2,\text{PLF}}=\sqrt{{\hat{\lambda }}_{2}^{2}+\frac{1}{2}\left(2{\hat{\lambda }}_{2}\sigma_{44}+A_{1}\sigma_{14}+A_{2}\sigma_{24}+A_{3}\sigma_{34}+A_{4}\sigma_{44}+A_{5}\sigma_{54}\right)}, \end{array}$$

(38) $$\begin{array}{c} \pi_{1,\text{PLF}}=\sqrt{{\hat{\pi }}_{1}^{2}+\frac{1}{2}\left(2{\hat{\pi }}_{1}\sigma_{55}+A_{1}\sigma_{15}+A_{2}\sigma_{25}+A_{3}\sigma_{35}+A_{4}\sigma_{45}+A_{5}\sigma_{55}\right)}. \end{array}$$

The BEs for the model parameters under ELF using NIP are

(39) $$\begin{array}{c} \theta_{1,\text{ELF}}={\left\{{\overset{\wedge }{\theta }}_{1}^{-1}+\frac{1}{2}\left(-{\overset{\wedge }{\theta }}_{1}^{-2}\sigma_{11}+A_{1}\sigma_{11}+A_{2}\sigma_{21}+A_{3}\sigma_{31}+A_{4}\sigma_{41}+A_{5}\sigma_{51}\right)\right\}}^{-1}, \end{array}$$

(40) $$\begin{array}{c} \theta_{2,\text{ELF}}={\left\{{\overset{\wedge }{\theta }}_{2}^{-1}+\frac{1}{2}\left(-{\overset{\wedge }{\theta }}_{2}^{-2}\sigma_{22}+A_{1}\sigma_{12}+A_{2}\sigma_{22}+A_{3}\sigma_{32}+A_{4}\sigma_{42}+A_{5}\sigma_{52}\right)\right\}}^{-1}, \end{array}$$

(41) $$\begin{array}{c} \lambda_{1,\text{ELF}}={\left\{{\overset{\wedge }{\lambda }}_{1}^{-1}+\frac{1}{2}\left(-{\overset{\wedge }{\lambda }}_{1}^{-2}\sigma_{33}+A_{1}\sigma_{13}+A_{2}\sigma_{23}+A_{3}\sigma_{33}+A_{4}\sigma_{43}+A_{5}\sigma_{53}\right)\right\}}^{-1}, \end{array}$$

(42) $$\begin{array}{c} \lambda_{2,\text{ELF}}={\left\{{\overset{\wedge }{\lambda }}_{2}^{-1}+\frac{1}{2}\left(-{\overset{\wedge }{\lambda }}_{2}^{-2}\sigma_{44}+A_{1}\sigma_{14}+A_{2}\sigma_{24}+A_{3}\sigma_{34}+A_{4}\sigma_{44}+A_{5}\sigma_{54}\right)\right\}}^{-1}, \end{array}$$

(43) $$\begin{array}{c} \pi_{1,\text{ELF}}={\left\{{\overset{\wedge }{\pi }}_{1}^{-1}+\frac{1}{2}\left(-{\overset{\wedge }{\pi }}_{1}^{-2}\sigma_{55}+A_{1}\sigma_{15}+A_{2}\sigma_{25}+A_{3}\sigma_{35}+A_{4}\sigma_{45}+A_{5}\sigma_{55}\right)\right\}}^{-1}. \end{array}$$

Finally, the BEs for the model parameters under LLF using NIP are

(44) $$\begin{array}{c} \theta_{1,\text{LLF}}=-\ln\left\{\exp\left(-{\hat{\theta }}_{1}\right)+\frac{1}{2}\left(-\exp\left(-{\hat{\theta }}_{1}\right)\sigma_{11}+A_{1}\sigma_{11}+A_{2}\sigma_{21}+A_{3}\sigma_{31}+A_{4}\sigma_{41}+A_{5}\sigma_{51}\right)\right\}, \end{array}$$

(45) $$\begin{array}{c} \theta_{2,\text{LLF}}=-\ln\left\{\exp\left(-{\hat{\theta }}_{2}\right)+\frac{1}{2}\left(-\exp\left(-{\hat{\theta }}_{2}\right)\sigma_{22}+A_{1}\sigma_{12}+A_{2}\sigma_{22}+A_{3}\sigma_{32}+A_{4}\sigma_{42}+A_{5}\sigma_{52}\right)\right\}, \end{array}$$

(46) $$\begin{array}{c} \lambda_{1,\text{LLF}}=-\ln\left\{\exp\left(-{\hat{\lambda }}_{1}\right)+\frac{1}{2}\left(-\exp\left(-{\hat{\lambda }}_{1}\right)\sigma_{33}+A_{1}\sigma_{13}+A_{2}\sigma_{23}+A_{3}\sigma_{33}+A_{4}\sigma_{43}+A_{5}\sigma_{53}\right)\right\}, \end{array}$$

(47) $$\begin{array}{c} \lambda_{2,\text{LLF}}=-\ln\left\{\exp\left(-{\hat{\lambda }}_{2}\right)+\frac{1}{2}\left(-\exp\left(-{\hat{\lambda }}_{2}\right)\sigma_{44}+A_{1}\sigma_{14}+A_{2}\sigma_{24}+A_{3}\sigma_{34}+A_{4}\sigma_{44}+A_{5}\sigma_{54}\right)\right\}, \end{array}$$

(48) $$\begin{array}{c} \pi_{1,\text{LLF}}=-\ln\left\{\exp\left(-{\hat{\pi }}_{1}\right)+\frac{1}{2}\left(-\exp\left(-{\hat{\pi }}_{1}\right)\sigma_{55}+A_{1}\sigma_{15}+A_{2}\sigma_{25}+A_{3}\sigma_{35}+A_{4}\sigma_{45}+A_{5}\sigma_{55}\right)\right\}. \end{array}$$

Similarly, for rest of the cases, the BEs for the parameters and RCs of the 2CMGED under right-censored samples can be obtained.

The article "On Suitability of Mixture of Generalized Exponential Models in Modeling Right-Censored Medical Datasets Using Conditional Expectations" was published in 2022. Journal: Comput Math Methods Med.

#### 2.1.4. Importance Sampling (IS)

In this section, the BEs for the parameters of 2CMGED have been considered using IS. For importance sampling, the first step is to identify the marginal and conditional densities from the posterior distribution. Interestingly in Equation (11), the parameter *π*_1_ follows beta distribution with parameters *r*_1_ + 1 and*r*_2_ + 1. On the other hand, the parameters *θ*_*j*_ have gamma distribution with parameters *r*_*j*_ + 1 and*κ*_1*j*_(*x*_*ji*_) = ∑_*i*=1_^*r*_*j*_^*x*_*ji*_. Similarly, the conditional distributions of *λ*_*j*_|*θ*_*j*_ are again gamma densities with parameters *r*_*j*_ + 1 and *χ*_1*j*_(*x*_*ji*_) = −∑_*i*=1_^*r*_*j*_^log(1 − *e*^−*θ*_*j*_*x*_*ji*_^), where *j* = 1, 2.Let

(49) $$\begin{array}{c} \begin{array}{c} h_{14}\left(\pi_{1},\theta_{j},\lambda_{j}\left|x\right.\right)={\left\{1-\pi_{1}{\left(1-e^{-\theta_{1}t}\right)}^{\lambda_{1}}-\left(1-\pi_{1}\right){\left(1-e^{-\theta_{1}t}\right)}^{\lambda_{2}}\right\}}^{n-r}\\ \times \exp\left\{-\overset{r_{1}}{\underset{i=1}{\sum }}\log\left(1-e^{-\theta_{1}x_{1i}}\right)\right\}\exp\left\{-\overset{r_{2}}{\underset{i=1}{\sum }}\log\left(1-e^{-\theta_{2}x_{2i}}\right)\right\}\overset{2}{\underset{j=1}{\prod }}{\left\{\kappa_{1j}\left(x_{ji}\right)\right\}}^{-r_{j}-1}{\left\{\chi_{1j}\left(x_{ji}\right)\right\}}^{-r_{j}-1}. \end{array} \end{array}$$

Now, the posterior distribution given in Equation (49) can be partitioned as follows:

(50) $$\begin{array}{c} g_{1}\left(\Omega \left|x\right.\right)\propto h_{11}\left(\pi_{1}\left|x\right.\right)h_{12}\left(\theta_{j}\left|x\right.\right)h_{13}\left(\lambda_{j}\left|\theta_{j},x\right.\right)h_{14}\left(\pi_{1},\lambda_{j},\theta_{j}\left|x\right.\right), \end{array}$$

where *π*_1_ ~ Beta(*r*_1_ + 1, *r*_2_ + 1), *θ*_*j*_ ~ Gamma(*r*_*j*_ + 1, *κ*_1*j*_(*x*_*ji*_)),

*λ*_*j*_|*θ*_*j*_ ~ Gamma(*r*_*j*_ + 1, *χ*_1*j*_(*x*_*ji*_))_,_ and *h*_14_(*π*_1_, *θ*_*j*_, *λ*_*j*_|**x**) are given in Equation (49).

Based on IS, the BEs for the parametric set **Ω**, under NIP using SELF, are

(51) $$\begin{array}{c} \pi_{1,\text{SELF}}=\frac{{Ε}^{\prime }\left[\pi_{1}h_{14}\left(\pi_{1},\theta_{j},\lambda_{j}\left|x\right.\right)\right]}{{Ε}^{\prime }\left[h_{14}\left(\pi_{1},\theta_{j},\lambda_{j}\left|x\right.\right)\right]},\;\theta_{j,\text{SELF}}=\frac{{Ε}^{\prime }\left[\theta_{j}h_{14}\left(\pi_{1},\theta_{j},\lambda_{j}\left|x\right.\right)\right]}{{Ε}^{\prime }\left[h_{14}\left(\pi_{1},\theta_{j},\lambda_{j}\left|x\right.\right)\right]},\;\lambda_{j,\text{SELF}}=\frac{{Ε}^{\prime }\left[\lambda_{j}h_{14}\left(\pi_{1},\theta_{j},\lambda_{j}\left|x\right.\right)\right]}{{Ε}^{\prime }\left[h_{14}\left(\pi_{1},\theta_{j},\lambda_{j}\left|x\right.\right)\right]}. \end{array}$$

For remaining cases, the similar methodology can be used for the estimation using IS.

## 3. Results and Discussions

In this subsection, the right-censored data have been generated from the 2CMGED for analysis. Based on these simulated data, the comparison among different estimators has been made with respect to various factors such as samples sizes, priors, LFs, and Bayesian approximation methods.

The article "On Suitability of Mixture of Generalized Exponential Models in Modeling Right-Censored Medical Datasets Using Conditional Expectations" was published in 2022. Journal: Comput Math Methods Med.

The steps for numerical simulations have been given in the followings:

*Step 1.* Generate a random sample of size ‘*n*' from the proposed model.

*Step 2.* Next generate uniformly distributed random number (*u*) corresponding to each value of the sample.

*Step 3.* The values of sample for *u* ≤ *π*_1_ have been considered to come from component-1 and the rest from component-2.

*Step 4.* Determine the censoring rate (Ri).

*Step 5.* The starting *n*—*n* × *Ri* values have been observed and remaining values have been assumed to be censored.

*Step 6.* Use the observed values for analysis.

*Step 7.* Repeat Step 1 to Step 6 10,000 times, and obtain the BEs using either LA or IS given in Subsections 2.1.3 and 2.1.4, respectively.

*Step 8.* Obtain the BEs by average of the results computed in Step 7.

Tables 1–12 and in Figures 1–10 contain the numerical and graphical results, respectively. The BEs for the parameters of the 2CMGED, under right-censored samples, have been presented in Tables 1–8. The performance of the posterior estimators has been investigated via amounts of associated PRs. From the results, it can be observed that larger samples sizes produced improved estimation for the model parameters. IPs and LLF come up with better estimation as compared to their counter parts. On the other hand, the estimates under IS seem better than those under LA with few exceptions. These trends are also observable from Figures 1–6.

Table 9 and Figure 9 capture the impact of change in mixing parameter (*π*_1_) on the estimation of 2CMGED. The samples of size 100 with 20% right censoring with *λ*_1_ = 0.50, *θ*_1_ = 1.20, *λ*_2_ = 0.75, *θ*_2_ = 1.50, and IP have been used for the estimation. The larger values of the mixing parameter improve the estimation for the first component of the 2CMGED with still reasonably good estimation for the second component of the 2CMGED. The effect of different censoring rates on the performance of the estimation from 2CMGED has been observed in Table 10 and in Figure 8. For estimation, we assumed *λ*_1_ = 0.50, *θ*_1_ = 1.20, *λ*_2_ = 0.75, *θ*_2_ = 1.50, *π*_1_ = 0.45, *n* = 100, LLF, and IP. As per expectations, the lower censoring rates provide the better estimation for the parameters of the 2CMGED. The results for different sets of the parametric values regarding right-censored 2CMGED have been reported in Table 11 and in Figure 10. The IP and LLF with 20% right-censored samples have been considered for this purpose. The smaller choices of the true parametric values from one component of 2CMGED result in improved estimation for the other component of the 2CMGED.

The article "On Suitability of Mixture of Generalized Exponential Models in Modeling Right-Censored Medical Datasets Using Conditional Expectations" was published in 2022. Journal: Comput Math Methods Med.

The estimation of the RCs from the right-censored 2CMGED has been given in Table 12. The estimation has been considered under 20% right-censored samples using *λ*_1_ = 0.50, *θ*_1_ = 1.20, *λ*_2_ = 0.75, *θ*_2_ = 1.50, *π*_1_ = 0.45, and *t* = 1.00 with *R*(*t*) = 0.1687, HR(*t*) = 1.4483, and RHR(*t*) = 0.2939. These RCs have been estimated using LA under different situations. The better estimation of the RCs has been observed for larger sample sizes. The advantage of using the IP with LLF has been seen in majority of cases.

Table 13 contains the comparison of results based on conventional censoring schemes and censoring schemes based on CE. From the results, it can be assessed that results based on CE-censored samples are superior to those under conventional censoring schemes. Similarly, Table 14 reports the impact of mixing parameter under CE-censored samples. The results in Table 14 are better than those under conventional censoring schemes given in Table 9. Further, comparing results reported in Table 10 (for conventional censoring schemes) and Table 15 (for CE based censoring schemes), the results under CE based censoring schemes were better irrespective of the choice of censoring rate. The results under conventional censoring schemes and CE based censoring schemes have also been compared for various choices of the true parametric values. The corresponding results have been reported in Table 11 and Table 16, respectively. These results elucidate that the CE-based censored samples provide improved estimation for the model parameters for different choices of the true parametric values.

### 3.1. Real Life Examples

In this section, two datasets regarding survival times for the cancer patients have been used to evaluate the applicability of the proposed model. The dataset-1 is about the survival times (in months) of 121 breast cancer patients. This dataset has been reported by Lawless. The (^∗^) denotes the censored times. The observations for the dataset-1 are as follows: 0.3, 0.3^∗^, 4.0^∗^, 5.0, 5.6, 6.2, 6.3, 6.6, 6.8, 7.4^∗^, 7.5, 8.4, 8.4, 10.3, 11.0, 11.8, 12.2, 12.3, 13.5, 14.4, 14.4, 14.8, 15.5^∗^, 15.7, 16.2, 16.3, 16.5, 16.8, 17.2, 17.3, 17.5, 17.9, 19.8, 20.4, 20.9, 21.0, 21.0, 21.1, 23.0, 23.4^∗^, 23.6, 24.0, 24.0, 27.9, 28.2, 29.1, 30, 31, 31, 32, 35, 35, 37^∗^, 37^∗^, 37^∗^, 38, 38^∗^, 38^∗^, 39^∗^, 39^∗^, 40, 40^∗^, 40^∗^, 41, 41, 41^∗^, 42, 43^∗^, 43^∗^, 43^∗^, 44 45^∗^, 45^∗^, 46^∗^, 46^∗^, 47^∗^, 48, 49^∗^, 51, 51, 51^∗^, 52, 54, 55^∗^, 56, 57^∗^, 58^∗^, 59^∗^, 60, 60, 60^∗^, 61^∗^, 62^∗^, 65^∗^, 65^∗^, 67^∗^, 67^∗^, 68^∗^, 69^∗^, 78, 80, 83^∗^, 88^∗^, 89, 90, 93^∗^, 96^∗^, 103, 105^∗^, 109^∗^, 109^∗^, 111^∗^, 115^∗^, 117^∗^, 125^∗^, 126, 127, 129^∗^, 129^∗^, 139^∗^, and 154^∗^. Out of 121 survival times, 56 are right censored. Therefore, the ratio of censoring in dataset-1 is around 46%.

The article "On Suitability of Mixture of Generalized Exponential Models in Modeling Right-Censored Medical Datasets Using Conditional Expectations" was published in 2022. Journal: Comput Math Methods Med.

The dataset-2 also reported by Lawless, contains the survival times (in days) of two groups of cancer patients. The first group contains 51 patients with head and neck cancer (HNC). This group was treated with radiotherapy (RT). The second group is comprised of 45 HNC patients treated with RT and chemotherapy (CT). The observations of both of these groups are as follows.

Group-I: 7, 34, 42, 63, 64, 74^∗^, 83, 84, 91, 108, 112, 129, 133, 133, 139, 140, 140, 146, 149, 154, 157, 160, 160, 165, 173, 176, 185^∗^, 218, 225, 241, 248, 273, 277, 279^∗^, 297, 319^∗^, 405, 417, 420, 440, 523, 523^∗^, 583, 594, 1101, 1116^∗^, 1146, 1226^∗^, 1349^∗^, 1412^∗^, and 1417.

Group-II: 37, 84, 92, 94, 110, 112, 119, 127, 130, 133, 140, 146, 155, 159, 169^∗^, 173, 179, 194, 195, 209, 249, 281, 319, 339, 432, 469, 519, 528^∗^, 547^∗^, 613^∗^, 633, 725, 759^∗^, 817, 1092^∗^, 1245^∗^, 1331^∗^, 1557^∗^, 1642^∗^, 1771^∗^, 1776, 1897^∗^, 2023^∗^, 2146^∗^, and 2297^∗^.

Out of 51 observations in group-I, 7 observations are right censored. So, in group-I, approximately 14% of the observations are right censored. On the other hand, in group-II, 15 out of 45 observations are right censored with censoring rate 33%. On the whole, for dataset-2, out of 96 observations 22 are right censored. Hence, for dataset-2, the censoring rate is approximately 23%. The descriptive statistics for dataset-1 and dataset-2 have been reported in Table 17. The results in Table 17 suggest that the real datasets used in the study are positively skewed and leptokurtic.

These data have been used to illustrate the applicability of the proposed model. The graphical display of goodness of fit for 2CMGED and 2CMED using dataset-1 and dataset-2 has been given in Figure 11. In particular, Figure 11(a) shows the comparison of empirical and theoretical densities for the competing models using dataset-1. Similarly, Figure 11(b) presents the comparison of empirical and theoretical CDFs for the competing models using dataset-1. On the other hand, Figure 11(c) and Figure 11(d) show the comparison of empirical and theoretical densities and CDFs for dataset-2, respectively. On the whole, Figure 11 suggests that the 2CMGED has better able to represent the behavior of both datasets as compared to 2CMED.

The modeling capabilities of the proposed model have been further evaluated using different goodness of fit criteria such as Akaike information criteria (AIC), Bayesian information criteria (BIC), Cramer-von Mises (CM) statistic, Anderson-Darling (AD) statistic, and Kolmogorov-Smirnov (KS) statistic. The results have been reported in Table 18. The results in Table 18 simply indicate that the results for all the goodness of fit statistics are smaller in case of 2CMGED and compared those for 2CMED. So, the performance of the 2CMGED is better as compared to 2CMED.

The article "On Suitability of Mixture of Generalized Exponential Models in Modeling Right-Censored Medical Datasets Using Conditional Expectations" was published in 2022. Journal: Comput Math Methods Med.

## 4. Conclusion

The study has been conducted to explore the suitability of 2CMGED to model the right-censored medical datasets having mixture behavior. In addition, the estimation of model parameters using CE-based censored samples has been introduced. The comparison of the results based on conventional and CE-based censored samples has also been reported. The Bayesian methods have been proposed to estimate the model parameters. In the first phase of the study, a detailed simulation study has been carried out to evaluate the performance of the proposed estimators. The numerical simulations have been carried out using R software. The results from the simulation study confirm the consistency property of the proposed estimators. The estimates based on IS, IP, and LLF were found superior to their counterparts. The results from the simulated study also advocate that the estimation using CE-based censored samples was superior to that under conventionally censored samples. The supremacy of CE-based censored samples was witnessed for different choices of sample size, true parametric values, mixing weights, and censoring rates. In second phase of the study, two real datasets relating to survival times of the cancer patients have been used to illustrate the applicability of the proposed model in medical field of study. In addition, the performance of the proposed 2CMGED was compared with 2CMED in molding said datasets. Based on various goodness of fit statistics such as AIC, BIC, CM statistic, AD statistic, and KS statistic, 2CMGED was found superior to 2CMED. Hence, 2CMGED was explored to be a very promising candidate for modeling survival times of the patients suffering from cancer.

Since the medical datasets can be left censored and doubly censored in some cases, the study can further be extended for the said censoring schemes. The study can also be extended for using lifetime models with bathtub shape hazard rates, because such models have been shown to fit the medical datasets efficiently.

## Figures and Tables

**Figure 1:** Graph for BEs using SELF NIP, and LA.

**Figure 2:** Graph for BEs using SELF, NIP, and IS.

**Figure 3:** Graph for PRs using SELF, NIP, and LA.

**Figure 4:** Graph for PRs using SELF, NP, and IS.

The article "On Suitability of Mixture of Generalized Exponential Models in Modeling Right-Censored Medical Datasets Using Conditional Expectations" was published in 2022. Journal: Comput Math Methods Med.

**Figure 5:** Comparison of BEs under IS and LA using NIF.

**Figure 6:** Comparison of LFs under LA and NIP.

**Figure 7:** Comparison of Priors using SELF and IS.

**Figure 8:** Effect on increase in CRs using ELF, IP, and IS.

**Figure 9:** Effect on increase in Pi using ELF, IP, and IS.

**Figure 10:** Effect of change in true parametric values.

**Figure 11:** Plots for empirical and theoretical densities and CDFs.

**Table 1:** Bayes estimation for the right-censored 2CMGED under SELF and NIP.

*n*	Technique	True parametric values				
		*λ*_1_ = 0.50	*θ*_1_ = 1.20	*λ*_2_ = 0.75	*θ*_2_ = 1.50	*π*_1_ = 0.45
20	LA	0.7076	1.6842	0.9767	2.3174	0.5895
		(0.0232)	(0.0609)	(0.0511)	(0.1813)	(0.0242)
	IS	0.7207	1.5813	1.0186	2.4312	0.6680
		(0.0050)	(0.0726)	(0.0094)	(0.1714)	(0.0051)
50	LA	0.6394	1.5216	0.8828	2.0937	0.5328
		(0.0165)	(0.0434)	(0.0367)	(0.1289)	(0.0173)
	IS	0.6535	1.4298	0.9236	2.1984	0.6056
		(0.0035)	(0.0519)	(0.0068)	(0.1233)	(0.0037)
100	LA	0.5748	1.3933	0.7663	1.8764	0.4790
		(0.0137)	(0.0373)	(0.0297)	(0.1084)	(0.0144)
	IS	0.5852	1.3066	0.7986	1.9662	0.5425
		(0.0030)	(0.0447)	(0.0054)	(0.1030)	(0.0030)
200	LA	0.5067	1.3588	0.7489	1.8483	0.4631
		(0.0085)	(0.0210)	(0.0161)	(0.0769)	(0.0075)
	IS	0.5194	1.2966	0.7770	1.8482	0.5227
		(0.0018)	(0.0265)	(0.0031)	(0.0845)	(0.0019)

**Table 2:** Bayes estimation for the right-censored 2CMGED under PLF and NIP.

*n*	Technique	True parametric values				
		*λ*_1_ = 0.50	*θ*_1_ = 1.20	*λ*_2_ = 0.75	*θ*_2_ = 1.50	*π*_1_ = 0.45
20	LA	0.7143	1.7041	0.9880	2.3252	0.5915
		(0.0409)	(0.1167)	(0.0982)	(0.1659)	(0.0360)
	IS	0.7276	1.5998	1.0304	2.4398	0.6702
		(0.0088)	(0.1400)	(0.0181)	(0.1583)	(0.0076)
50	LA	0.6455	1.5394	0.8931	2.1008	0.5346
		(0.0294)	(0.0838)	(0.0699)	(0.1192)	(0.0257)
	IS	0.6595	1.4465	0.9342	2.2060	0.6076
		(0.0063)	(0.1003)	(0.0128)	(0.1131)	(0.0054)
100	LA	0.5802	1.4098	0.7749	1.8827	0.4806
		(0.0246)	(0.0714)	(0.0566)	(0.0995)	(0.0214)
	IS	0.5907	1.3218	0.8078	1.9730	0.5443
		(0.0053)	(0.0859)	(0.0104)	(0.0946)	(0.0046)
200	LA	0.5105	1.3645	0.7538	1.8768	0.4670
		(0.0180)	(0.0471)	(0.0308)	(0.0507)	(0.0128)
	IS	0.5234	1.3019	0.7820	1.8764	0.5271
		(0.0037)	(0.0594)	(0.0055)	(0.0556)	(0.0033)

**Table 3:** Bayes estimation for the right-censored 2CMGED under LLF and NIP.

*n*	Technique	True parametric values				
		*λ*_1_ = 0.50	*θ*_1_ = 1.20	*λ*_2_ = 0.75	*θ*_2_ = 1.50	*π*_1_ = 0.45
20	LA	0.6838	1.6215	0.9382	2.2382	0.5736
		(0.0180)	(0.0484)	(0.0406)	(0.1486)	(0.0194)
	IS	0.6945	1.5215	0.9889	2.3601	0.6432
		(0.0038)	(0.0562)	(0.0076)	(0.1371)	(0.0041)
50	LA	0.6182	1.4634	0.8579	2.0170	0.5160
		(0.0132)	(0.0338)	(0.0294)	(0.0993)	(0.0139)
	IS	0.6297	1.3915	0.8954	2.1316	0.5860
		(0.0028)	(0.0406)	(0.0054)	(0.0958)	(0.0029)
100	LA	0.5560	1.3422	0.7410	1.8267	0.4628
		(0.0108)	(0.0280)	(0.0236)	(0.0871)	(0.0112)
	IS	0.5664	1.2580	0.7741	1.9011	0.5254
		(0.0023)	(0.0362)	(0.0041)	(0.0831)	(0.0024)
200	LA	0.4901	1.3212	0.7227	1.8004	0.4454
		(0.0066)	(0.0169)	(0.0130)	(0.0628)	(0.0060)
	IS	0.5033	1.2638	0.7549	1.7859	0.5087
		(0.0015)	(0.0207)	(0.0024)	(0.0678)	(0.0015)

The article "On Suitability of Mixture of Generalized Exponential Models in Modeling Right-Censored Medical Datasets Using Conditional Expectations" was published in 2022. Journal: Comput Math Methods Med.

**Table 4:** Bayes estimation for the right-censored 2CMGED under ELF and NIP.

*n*	Technique	True parametric values				
		*λ*_1_ = 0.50	*θ*_1_ = 1.20	*λ*_2_ = 0.75	*θ*_2_ = 1.50	*π*_1_ = 0.45
20	LA	0.6904	1.6353	0.9522	2.2791	0.5739
		(0.0216)	(0.0575)	(0.0471)	(0.1676)	(0.0228)
	IS	0.7095	1.5349	0.9903	2.3689	0.6501
		(0.0046)	(0.0683)	(0.0088)	(0.1584)	(0.0048)
50	LA	0.6262	1.4935	0.8624	2.0479	0.5233
		(0.0153)	(0.0403)	(0.0343)	(0.1221)	(0.0164)
	IS	0.6387	1.3940	0.8995	2.1403	0.5900
		(0.0032)	(0.0482)	(0.0064)	(0.1129)	(0.0035)
100	LA	0.5617	1.3659	0.7532	1.8235	0.4668
		(0.0127)	(0.0347)	(0.0280)	(0.1011)	(0.0133)
	IS	0.5730	1.2798	0.7788	1.9146	0.5333
		(0.0028)	(0.0410)	(0.0051)	(0.0964)	(0.0028)
200	LA	0.4926	1.3308	0.7351	1.8197	0.4524
		(0.0079)	(0.0199)	(0.0147)	(0.0727)	(0.0070)
	IS	0.5115	1.2749	0.7653	1.8161	0.5132
		(0.0016)	(0.0250)	(0.0028)	(0.0784)	(0.0018)

**Table 5:** Bayes estimation for the right-censored 2CMGED under SELF and IP.

*n*	Technique	True parametric values				
		*λ*_1_ = 0.50	*θ*_1_ = 1.20	*λ*_2_ = 0.75	*θ*_2_ = 1.50	*π*_1_ = 0.45
20	LA	0.6837	1.6264	0.9439	2.2377	0.5697
		(0.0211)	(0.1433)	(0.0473)	(0.1693)	(0.0222)
	IS	0.6970	1.5291	0.9848	2.3509	0.6459
		(0.0045)	(0.1713)	(0.0087)	(0.1601)	(0.0047)
50	LA	0.6189	1.4717	0.8542	2.0248	0.5155
		(0.0152)	(0.1024)	(0.0336)	(0.1207)	(0.0159)
	IS	0.6345	1.3859	0.8968	2.1310	0.5880
		(0.0033)	(0.1226)	(0.0060)	(0.1145)	(0.0033)
100	LA	0.5591	1.4467	0.7985	1.8314	0.4659
		(0.0125)	(0.0847)	(0.0269)	(0.1010)	(0.0131)
	IS	0.5695	1.3579	0.8326	1.9211	0.5279
		(0.0028)	(0.1016)	(0.0049)	(0.0960)	(0.0029)
200	LA	0.4936	1.3577	0.7482	1.8083	0.4615
		(0.0078)	(0.0474)	(0.0149)	(0.0714)	(0.0068)
	IS	0.5067	1.2957	0.7852	1.8086	0.5217
		(0.0016)	(0.0608)	(0.0027)	(0.0781)	(0.0019)

**Table 6:** Bayes estimation for the right-censored 2CMGED under PLF and IP.

*n*	Technique	True parametric values				
		*λ*_1_ = 0.50	*θ*_1_ = 1.20	*λ*_2_ = 0.75	*θ*_2_ = 1.50	*π*_1_ = 0.45
20	LA	0.6903	1.6456	0.9549	2.2454	0.5716
		(0.0378)	(0.1073)	(0.0904)	(0.1522)	(0.0332)
	IS	0.7036	1.5470	0.9962	2.3592	0.6482
		(0.0081)	(0.1287)	(0.0165)	(0.1448)	(0.0070)
50	LA	0.6246	1.4891	0.8641	2.0319	0.5172
		(0.0271)	(0.0768)	(0.0644)	(0.1096)	(0.0236)
	IS	0.6405	1.4022	0.9072	2.1382	0.5901
		(0.0057)	(0.0920)	(0.0118)	(0.1034)	(0.0050)
100	LA	0.5645	1.4346	0.7808	1.8377	0.4675
		(0.0224)	(0.0653)	(0.0517)	(0.0911)	(0.0196)
	IS	0.5748	1.3463	0.8142	1.9276	0.5296
		(0.0048)	(0.0779)	(0.0094)	(0.0867)	(0.0041)
200	LA	0.4973	1.3632	0.7525	1.8359	0.4549
		(0.0163)	(0.0429)	(0.0277)	(0.0462)	(0.0118)
	IS	0.5106	1.2848	0.7903	1.8361	0.5143
		(0.0033)	(0.0539)	(0.0051)	(0.0508)	(0.0031)

The article "On Suitability of Mixture of Generalized Exponential Models in Modeling Right-Censored Medical Datasets Using Conditional Expectations" was published in 2022. Journal: Comput Math Methods Med.

**Table 7:** Bayes estimation for the right-censored 2CMGED under LLF and IP.

*n*	Technique	True parametric values				
		*λ*_1_ = 0.50	*θ*_1_ = 1.20	*λ*_2_ = 0.75	*θ*_2_ = 1.50	*π*_1_ = 0.45
20	LA	0.6607	1.5658	0.9067	2.1613	0.5544
		(0.0164)	(0.1138)	(0.0376)	(0.1388)	(0.0178)
	IS	0.6717	1.4713	0.9561	2.2821	0.6219
		(0.0034)	(0.1326)	(0.0071)	(0.1281)	(0.0037)
50	LA	0.5984	1.4154	0.8301	1.9506	0.4993
		(0.0121)	(0.0798)	(0.0269)	(0.0929)	(0.0128)
	IS	0.6113	1.3488	0.8694	2.0662	0.5690
		(0.0027)	(0.0960)	(0.0047)	(0.0890)	(0.0026)
100	LA	0.5408	1.3937	0.7721	1.7829	0.4502
		(0.0098)	(0.0636)	(0.0213)	(0.0812)	(0.0102)
	IS	0.5512	1.3074	0.8070	1.8575	0.5113
		(0.0022)	(0.0823)	(0.0037)	(0.0774)	(0.0024)
200	LA	0.4774	1.3202	0.7220	1.7615	0.4439
		(0.0061)	(0.0381)	(0.0120)	(0.0583)	(0.0054)
	IS	0.4910	1.2629	0.7628	1.7477	0.5078
		(0.0013)	(0.0474)	(0.0021)	(0.0627)	(0.0015)

**Table 8:** Bayes estimation for the right-censored 2CMGED under ELF and IP.

*n*	Technique	True parametric values				
		*λ*_1_ = 0.50	*θ*_1_ = 1.20	*λ*_2_ = 0.75	*θ*_2_ = 1.50	*π*_1_ = 0.45
20	LA	0.6671	1.5792	0.9202	2.2008	0.5546
		(0.0196)	(0.1352)	(0.0436)	(0.1565)	(0.0209)
	IS	0.6861	1.4842	0.9574	2.2906	0.6286
		(0.0041)	(0.1612)	(0.0081)	(0.1480)	(0.0045)
50	LA	0.6061	1.4445	0.8345	1.9805	0.5063
		(0.0141)	(0.0950)	(0.0314)	(0.1143)	(0.0150)
	IS	0.6201	1.3512	0.8734	2.0747	0.5728
		(0.0030)	(0.1138)	(0.0057)	(0.1048)	(0.0031)
100	LA	0.5464	1.4183	0.7849	1.7798	0.4540
		(0.0116)	(0.0788)	(0.0254)	(0.0942)	(0.0121)
	IS	0.5576	1.3301	0.8119	1.8707	0.5190
		(0.0026)	(0.0931)	(0.0046)	(0.0898)	(0.0027)
200	LA	0.4798	1.3298	0.7344	1.7804	0.4508
		(0.0073)	(0.0449)	(0.0136)	(0.0675)	(0.0063)
	IS	0.4990	1.2740	0.7733	1.7772	0.5123
		(0.0015)	(0.0573)	(0.0025)	(0.0725)	(0.0018)

**Table 9:** Effect of mixing parameter on the estimation of right-censored 2CMGED using LLF and IP.

*π*	Technique	Estimated values of the parameters				
		*λ*_1_	*θ*_1_	*λ*_2_	*θ*_2_	*π*_1_
0.25	LA	0.6067	1.5648	0.7738	1.7655	0.2303
		(0.0131)	(0.0905)	(0.0246)	(0.0923)	(0.0056)
	IS	0.6264	1.4839	0.7905	1.8121	0.2641
		(0.0029)	(0.1055)	(0.0046)	(0.0877)	(0.0012)
0.50	LA	0.5398	1.4013	0.7912	1.7940	0.4858
		(0.0115)	(0.0779)	(0.0256)	(0.0949)	(0.0129)
	IS	0.5509	1.3141	0.8184	1.8857	0.5553
		(0.0026)	(0.0920)	(0.0047)	(0.0905)	(0.0029)
0.75	LA	0.5213	1.3841	0.8468	1.9666	0.7150
		(0.0108)	(0.0730)	(0.0299)	(0.1082)	(0.0190)
	IS	0.5385	1.2865	0.8851	2.0706	0.8089
		(0.0024)	(0.0860)	(0.0054)	(0.1036)	(0.0043)

The article "On Suitability of Mixture of Generalized Exponential Models in Modeling Right-Censored Medical Datasets Using Conditional Expectations" was published in 2022. Journal: Comput Math Methods Med.

**Table 10:** Effect of censoring rates on the estimation of right-censored 2CMGED using LLF and IP.

CR	Technique	Estimated values of the parameters				
		*λ*_1_	*θ*_1_	*λ*_2_	*θ*_2_	*π*_1_
10%	LA	0.5326	1.3940	0.7829	1.7484	0.4496
		(0.0114)	(0.0751)	(0.0245)	(0.0908)	(0.0116)
	IS	0.5473	1.3130	0.8079	1.8345	0.5170
		(0.0024)	(0.0904)	(0.0045)	(0.0860)	(0.0026)
20%	LA	0.5464	1.4183	0.7849	1.7798	0.4540
		(0.0116)	(0.0788)	(0.0254)	(0.0942)	(0.0121)
	IS	0.5576	1.3301	0.8119	1.8707	0.5190
		(0.0026)	(0.0931)	(0.0046)	(0.0898)	(0.0027)
30%	LA	0.5671	1.5033	0.8289	1.8724	0.4788
		(0.0132)	(0.0902)	(0.0289)	(0.1061)	(0.0135)
	IS	0.5851	1.4212	0.8476	1.9704	0.5546
		(0.0029)	(0.1055)	(0.0052)	(0.1012)	(0.0030)

**Table 11:** Effect of true parametric values on the estimation using LLF and IP.

(*λ*_1_, *θ*_1_, *λ*_2_, *θ*_2_, *π*_1_)	Technique	Estimated values of the parameters				
		*λ*_1_	*θ*_1_	*λ*_2_	*θ*_2_	*π*_1_
(0.50, 1.20, 0.75, 1.50, 0.45)	LA	0.5464	1.4183	0.7849	1.7798	0.4540
		(0.0116)	(0.0788)	(0.0254)	(0.0942)	(0.0121)
	IS	0.5576	1.3301	0.8119	1.8707	0.5190
		(0.0026)	(0.0931)	(0.0046)	(0.0898)	(0.0027)
(0.50, 1.20, 1.50, 3.00, 0.45)	LA	0.5501	1.3929	1.5196	3.4386	0.4515
		(0.0130)	(0.0904)	(0.0674)	(0.3010)	(0.0126)
	IS	0.5505	1.3244	1.6161	3.5367	0.5115
		(0.0029)	(0.1065)	(0.0246)	(0.3395)	(0.0026)
(1.00, 2.40, 0.75, 1.50, 0.45)	LA	1.0401	2.7969	0.7727	1.7948	0.4625
		(0.0284)	(0.2511)	(0.0273)	(0.0977)	(0.0126)
	IS	1.0420	2.5988	0.8432	1.8419	0.5294
		(0.0063)	(0.3002)	(0.0049)	(0.0946)	(0.0024)

**Table 12:** BEs for RCs of the right-censored 2CMGED.

*n*	Loss function	NIP			IP		
		*R*(*t*)	HR(*t*)	RHR(*t*)	*R*(*t*)	HR(*t*)	RHR(*t*)
20	SELF	0.1118	2.0554	0.3418	0.1148	2.0439	0.3303
		(0.0209)	(0.3815)	(0.0278)	(0.0193)	(0.3510)	(0.0257)
	PLF	0.1128	2.0669	0.3429	0.1160	2.0554	0.3315
		(0.0266)	(0.2943)	(0.0345)	(0.0245)	(0.2708)	(0.0318)
	ELF	0.1091	1.9957	0.3332	0.1129	1.9899	0.3223
		(0.0194)	(0.3599)	(0.0256)	(0.0178)	(0.3312)	(0.0240)
	LLF	0.1090	1.9899	0.3294	0.1120	2.0001	0.3201
		(0.0206)	(0.2337)	(0.0274)	(0.0201)	(0.2175)	(0.0254)

50	SELF	0.1198	1.9375	0.3247	0.1207	1.9272	0.3141
		(0.0136)	(0.2106)	(0.0252)	(0.0125)	(0.1930)	(0.0232)
	PLF	0.1211	1.9486	0.3258	0.1230	1.9382	0.3153
		(0.0172)	(0.1603)	(0.0309)	(0.0156)	(0.1469)	(0.0283)
	ELF	0.1179	1.8806	0.3157	0.1176	1.8756	0.3062
		(0.0125)	(0.1981)	(0.0236)	(0.0116)	(0.1831)	(0.0217)
	LLF	0.1171	1.8741	0.3166	0.1185	1.8772	0.3047
		(0.0137)	(0.1249)	(0.0247)	(0.0120)	(0.1181)	(0.0224)

100	SELF	0.1391	1.6396	0.3164	0.1427	1.6168	0.3065
		(0.0088)	(0.1157)	(0.0228)	(0.0078)	(0.1059)	(0.0209)
	PLF	0.1463	1.6606	0.3303	0.1500	1.6428	0.3201
		(0.0130)	(0.0975)	(0.0264)	(0.0120)	(0.0892)	(0.0242)
	ELF	0.1362	1.6093	0.3091	0.1396	1.5881	0.3002
		(0.0082)	(0.1074)	(0.0213)	(0.0074)	(0.1002)	(0.0196)
	LLF	0.1415	1.5997	0.3194	0.1460	1.5873	0.3097
		(0.0102)	(0.0732)	(0.0209)	(0.0096)	(0.0693)	(0.0189)

200	SELF	0.1578	1.4922	0.3067	0.1618	1.4867	0.2944
		(0.0063)	(0.0879)	(0.0210)	(0.0058)	(0.0801)	(0.0188)
	PLF	0.1609	1.4984	0.3056	0.1630	1.4928	0.2934
		(0.0079)	(0.0667)	(0.0254)	(0.0073)	(0.0607)	(0.0228)
	ELF	0.1554	1.4673	0.3021	0.1590	1.4598	0.2895
		(0.0058)	(0.0828)	(0.0193)	(0.0054)	(0.0747)	(0.0174)
	LLF	0.1559	1.4605	0.2969	0.1575	1.4529	0.2849
		(0.0064)	(0.0520)	(0.0195)	(0.0059)	(0.0490)	(0.0181)

The article "On Suitability of Mixture of Generalized Exponential Models in Modeling Right-Censored Medical Datasets Using Conditional Expectations" was published in 2022. Journal: Comput Math Methods Med.

**Table 13:** Comparison of estimates under conventional and CE censoring using ELF, IP, and IS.

*n*	Technique	True parametric values					KS Statistic	*P* value
		*λ*_1_ = 0.50	*θ*_1_ = 1.20	*λ*_2_ = 0.75	*θ*_2_ = 1.50	*π*_1_ = 0.45		
20	Conventional	0.6861	1.4842	0.9574	2.2906	0.6286	0.1689	0.7631
		(0.0041)	(0.1612)	(0.0081)	(0.1480)	(0.0045)		
	CE	0.6450	1.4337	0.9283	2.1584	0.6018	0.1579	0.7926
		(0.0036)	(0.1401)	(0.0072)	(0.1334)	(0.0040)		
50	Conventional	0.6201	1.3512	0.8734	2.0747	0.5728	0.1518	0.8065
		(0.0030)	(0.1138)	(0.0057)	(0.1048)	(0.0031)		
	CE	0.5812	1.3305	0.8641	1.9455	0.5399	0.1402	0.8627
		(0.0027)	(0.1012)	(0.0051)	(0.0913)	(0.0028)		
100	Conventional	0.5576	1.3301	0.8119	1.8707	0.5190	0.1331	0.8886
		(0.0026)	(0.0931)	(0.0046)	(0.0898)	(0.0027)		
	CE	0.5203	1.3041	0.7917	1.7090	0.4970	0.1326	0.9141
		(0.0023)	(0.0807)	(0.0041)	(0.0776)	(0.0024)		
200	Conventional	0.4990	1.2740	0.7733	1.7772	0.5123	0.0864	0.9370
		(0.0015)	(0.0573)	(0.0025)	(0.0725)	(0.0018)		
	CE	0.5028	1.2124	0.7508	1.5878	0.4915	0.0624	0.9684
		(0.0014)	(0.0494)	(0.0021)	(0.0634)	(0.0016)		

**Table 14:** Effect of mixing parameter on the estimation based on CE-censored samples using LLF and IP.

*π*	Technique	Estimated values of the parameters				
		*λ*_1_	*θ*_1_	*λ*_2_	*θ*_2_	*π*_1_
0.25	LA	0.5917	1.5295	0.7558	1.7140	0.2435
		(0.0109)	(0.0792)	(0.0203)	(0.0757)	(0.0049)
	IS	0.6096	1.4510	0.7684	1.7752	0.2579
		(0.0024)	(0.0927)	(0.0038)	(0.0717)	(0.0011)
0.50	LA	0.5280	1.3676	0.7709	1.7448	0.4906
		(0.0096)	(0.0684)	(0.0212)	(0.0779)	(0.0113)
	IS	0.5353	1.2789	0.7945	1.8342	0.5441
		(0.0022)	(0.0806)	(0.0039)	(0.0741)	(0.0026)
0.75	LA	0.5074	1.3492	0.8227	1.9146	0.7204
		(0.0090)	(0.0643)	(0.0247)	(0.0887)	(0.0166)
	IS	0.5253	1.2591	0.8618	2.0108	0.7927
		(0.0020)	(0.0752)	(0.0045)	(0.0852)	(0.0038)

**Table 15:** Effect of censoring rates on the estimation CE-censored samples using LLF and IP.

CR	Technique	Estimated values of the parameters				
		*λ*_1_	*θ*_1_	*λ*_2_	*θ*_2_	*π*_1_
10%	LA	0.5194	1.3597	0.7629	1.7084	0.4387
		(0.0094)	(0.0658)	(0.0203)	(0.0742)	(0.0102)
	IS	0.5317	1.2862	0.7914	1.7962	0.5061
		(0.0020)	(0.0791)	(0.0037)	(0.0703)	(0.0023)
20%	LA	0.5342	1.3874	0.7637	1.7414	0.4404
		(0.0096)	(0.0689)	(0.0210)	(0.0774)	(0.0106)
	IS	0.5434	1.2976	0.7888	1.8146	0.5045
		(0.0022)	(0.0819)	(0.0038)	(0.0739)	(0.0024)
30%	LA	0.5543	1.4677	0.8060	1.8331	0.4677
		(0.0110)	(0.0794)	(0.0240)	(0.0869)	(0.0118)
	IS	0.5700	1.3871	0.8272	1.9276	0.5415
		(0.0024)	(0.0924)	(0.0043)	(0.0827)	(0.0026)

The article "On Suitability of Mixture of Generalized Exponential Models in Modeling Right-Censored Medical Datasets Using Conditional Expectations" was published in 2022. Journal: Comput Math Methods Med.

**Table 16:** Effect of true parametric values on estimation based on CE-censored samples using LLF and IP.

(*λ*_1_, *θ*_1_, *λ*_2_, *θ*_2_, *π*_1_)	Technique	Estimated values of the parameters				
		*λ*_1_	*θ*_1_	*λ*_2_	*θ*_2_	*π*_1_
(0.50, 1.20, 0.75, 1.50, 0.45)	LA	0.5317	1.3838	0.7690	1.7322	0.4601
		(0.0097)	(0.0692)	(0.0211)	(0.0772)	(0.0107)
	IS	0.5437	1.3032	0.7923	1.8199	0.5061
		(0.0021)	(0.0814)	(0.0038)	(0.0732)	(0.0024)
(0.50, 1.20, 1.50, 3.00, 0.45)	LA	0.5376	1.3617	1.4876	3.3375	0.4560
		(0.0108)	(0.0797)	(0.0561)	(0.2473)	(0.0111)
	IS	0.5385	1.2868	1.5829	3.4357	0.5009
		(0.0024)	(0.0939)	(0.0204)	(0.2786)	(0.0023)
(1.00, 2.40, 0.75, 1.50, 0.45)	LA	1.0189	2.7294	0.7550	1.7482	0.4516
		(0.0235)	(0.2214)	(0.0225)	(0.0800)	(0.0111)
	IS	1.0144	2.5426	0.8226	1.7980	0.5158
		(0.0052)	(0.2626)	(0.0041)	(0.0775)	(0.0021)

**Table 17:** Descriptive statistics for real datasets.

Data	Mean	Median	Variance	Standard deviation	Skewness	Kurtosis
Dataset-1	32.30	22.05	772.21	27.79	1.68	5.66
Dataset-2 (group-I)	280.17	160.00	91884.73	303.12	2.32	8.10
Dataset-2 (group-II)	304.90	176.00	116532.10	341.37	2.94	12.66

**Table 18:** Goodness of fit statistics for real datasets.

Dataset	Model	AIC	BIC	CM statistic	AD statistic	KS statistic	*P* value (KS statistic)
Dataset-1	2CMGED	563.5029	574.3748	0.0684	0.4470	0.0883	0.9835
	2CMED	570.6215	577.1447	0.4232	2.5252	0.1564	0.8286
Dataset-2	2CMGED	276.0819	287.2524	0.0220	0.1781	0.0405	0.9241
	2CMED	294.1407	300.8430	0.3717	2.1951	0.1570	0.6124

## Data Availability

The data used in the paper are available in the paper.

## Abbreviations

2CMED: Two-component mixture of exponential distribution
2CMGED: Two-component mixture of generalized exponential distribution
AD: Anderson-Darling
AIC: Akaike information criteria
BEs: Bayes estimates
BIC: Bayesian information criteria
CDF: Cumulative distribution function
CE: Conditional expectations
CM: Cramer-von Mises
CT: Chemotherapy
ECDF: Empirical cumulative distribution function
ELF: Entropy loss function
HNC: Head and neck cancer
IP: Informative prior
IS: Importance sampling
KS: Kolmogorov-Smirnov
LA: Lindley's approximation
LLF: LINEX loss function
NIP: Noninformative prior
PLF: Precautionary loss function
RCs: Reliability characteristics
RT: Radiotherapy
SELF: Squared Error Loss Function.
